The article "Éclaircissement to Understand Consumers’ Decision-Making Psyche and Gender Effects, a Fuzzy Set Qualitative Comparative Analysis" was retracted in 2025. Reasons: unreliable results or conclusions; a conflict of interest; concerns about the peer review; concerns about the citations.

# Éclaircissement to Understand Consumers’ Decision-Making Psyche and Gender Effects, a Fuzzy Set Qualitative Comparative Analysis

**DOI:** 10.3389/fpsyg.2022.920594

**Published:** 2022-06-02

**Authors:** Sohaib Mustafa, Muhammad Tayyab Sohail, Roobaea Alroobaea, Saeed Rubaiee, A. Anas, Asem Majed Othman, Muhammad Nawaz

**Affiliations:** ^1^College of Economics and Management, Beijing University of Technology, Beijing, China; ^2^South Asian Research Centre, School of Public Administration, Xiangtan University, Xiangtan, China; ^3^Department of Computer Science, College of Computers and Information Technology, Taif University, Taif, Saudi Arabia; ^4^Department of Industrial and Systems Engineering, College of Engineering, University of Jeddah, Jeddah, Saudi Arabia; ^5^Department of Mechanical and Materials Engineering, College of Engineering, University of Jeddah, Jeddah, Saudi Arabia; ^6^Department of Business Administration, National College of Business Administration and Economics, Lahore, Pakistan

**Keywords:** consumer decision-making, fuzzy set qualitative comparative analysis (*fs*QCA), configurations, smartwatches, gender-specific psyche, UTAUT, use behavior, gender-difference in purchase

## Abstract

Consumers’ decision-making is complex and diverse in terms of gender. Different social, psychological, and economic factors mold the decision-making preferences of consumers. Most researchers used a variance-based approach to explain consumer decision-making that assumes symmetric relationship between variables. We have collected data from 468 smartwatch users and applied a fuzzy set qualitative comparative analysis (*fs*QCA) to explain and compare male and female consumers’ decision-making complexity. *f*sQCA assumes that an asymmetric relationship between variables can exist in the real world, and different combinations of variables can lead to the same output. Results explain that different variables have a core and secondary level of impact on consumer decision-making. Hence, we can not claim that certain factors are significant or insignificant for decision-making. *fs*QCA results revealed that cost value, performance expectancy, and social influence play a key role in consumers’ buying decisions. This study has contributed to the existing literature by explaining consumer decision-making by applying configuration and complexity theories and identifying unique solutions for both genders. A major contribution to theoretical literature was also made by this research, which revealed the complexity of consumer purchasing decisions made for new products.

## Introduction

The consumer electronics industry’s area of wearable electronic gadgets has grown rapidly. Despite humans having worn clocks for generations, the newest gadgets use cutting-edge mobile technology and do much more than merely tell the time. In addition to serving as fashion pieces, fitness trackers, gaming gadgets, and navigation aids, wearables come in various shapes and sizes. In terms of communication and health monitoring on the move, a smartwatch (SW), a small gadget worn around the wrist, has a smartphone’s capabilities virtually. As the next generation of consumer electronics, smartwatches are expected to alter consumers’ daily lives.

First to market with smartwatches (SWs) were Samsung, Sony, and LG. With the introduction of the iWatch, Apple made its first foray into the disruptive smartwatch business and quickly rose to the top of the chain. Apple, Samsung, Fitbit, Lenovo, Garmin, Huawei are the leading companies producing smartwatches.

The SWs feature a wide range of functions, including internet access, phone calls, weather updates, text and video communications, GPS navigation, and health and fitness data. It also has a touch screen interface and management apps similar to smartphones.

From 37 million in 2016 to over 258 million in 2025, the global shipments of smartwatches are expected to expand rapidly^1^. From 2019 to 2022, global shipments of wearable gadgets are estimated to double^1^. The worldwide smartwatch industry is predicted to be worth USD 57.3 billion in 2021. By 2026, it is expected to reach USD 132.9 Billion. An annual compound growth rate of about 18.32% throughout the predicted timeframe^2^. The three major smartwatch manufacturers have effectively infiltrated the conventional watch market’s mid-price category in the United States to get to the top of the watch best-seller list. In addition, smartwatch dollar sales increased by 51% in 2018, and smartwatch unit sales increased by 61%, according to NPD^3^. According to Brack^2^, SWs sold 55% more over the Christmas season in 2018 than regular watches did. SW’s market share is predicted to rise to USD 81 million by 2021 in the overall wearable market (Mokhtari et al., 2020).

The decision-making process of consumers is a complicated phenomenon (Brown and Venkatesh, 2005). Customers’ adoption of new items or technology is unquestionably influenced by social, economic, intrinsic, and psychological factors. These factors play an important role in consumers’ buying decisions (Mustafa et al., 2022). According to our best knowledge, no research has been undertaken on the different factors affecting consumers’ decision to purchase SWs. Furthermore, no study has exclusively generated gender-specific solutions to understand smartwatches’ buying behavior of different genders. Thus, empirical research into the factors affecting a user’s choice to purchase SWs is crucial. It will benefit our understanding of consumer decision-making about the purchase of SWs and enable SW producing companies to develop effective market strategies.

To a significant degree, research on technology adoption use approaches from the 1st or 2nd generations of multivariate models (e.g., multiple regression). It assumes that variables have symmetric relationships (e.g., SEM) (De Kervenoael et al., 2021). Predictors, in these models, are required to be both adequate and necessary for an event to take place. When symmetrical links between variables are assumed, a single optimal solution that precisely depicts the outcome may be shown to be the best option. There is a risk in placing too much emphasis on symmetric correlations since these effects precisely may not be present in datasets.

However, as is the case in real life, the interactions between variables in a dataset are exceedingly complex and are not always symmetrical or balanced (Woodside, 2017). Consequently, it is very unlikely that the two variables will have a symmetrical connection (Ragin, 2008; Woodside, 2014). For instance, effort expectation may be sufficient to justify a purchase. However, people may be content even if the product falls short of their expectations for effort or perceived performance, as long as they have a nice experience. Consequently, effort or perceived expectancy may not be required to achieve the expected results, signaling the need for a novel approach to identifying asymetric connections.

Previous studies (Alam et al., 2020; Gul et al., 2021; Awan et al., 2022; Jamil et al., 2022) study the consumer decision making assuming that variables have symmetric relationships. Whereas researchers such as (Ragin, 2008; Woodside, 2014) claim that its unlikely to have a symmetric relationship between the variables. Researchers have also claimed that multivariate models do not have the capacity to capture the asymmetric relationship between variables because these models count for single net effect of relationship. As consumer decision-making process is complex hence there is a need to utilize the novel methodology that emphasizes the interaction between variables and proposed to study the complex asymmetric relationships between variables (Ragin, 2008; Woodside, 2014).

Hence, asymmetric and symmetric analytical techniques are used in this study to evaluate and explore the interrelationships between the causes of behavior and the behavior of smartwatch users in order to fill in the research gaps previously highlighted. The fuzzy set qualitative comparative analysis (*fs*QCA) is a regularly used asymmetric approach that uncovers patterns in data that are generally hidden by symmetric methods (Sahibzada et al., 2020b). *fs*QCA findings will give a more comprehensive model for management that will assist identify the causal recipes that can successfully lead to better outcomes (Sahibzada et al., 2020a). Smartwatches manufacturing companies should be able to determine ways to improve their customers’ degree of use behavior since human decision-making is a complex phenomenon (Brown and Venkatesh, 2005). There are several aspects that influence smartwatch use that must be examined, and this can only be done with the help of *fs*QCA.

The suggested methodology brings theoretical and methodological advances to the research of human decision making psychology. Theoretically, the research is valid

1. Demonstrates the importance of decision making variables in influencing customer use behavior and decision making by analyzing the influence of each of the many aspects of decision making factors.
2. Brings more insight into current theories and paradigms such as UTAUT (Venkatesh et al., 2003), UTAUT2 (Venkatesh et al., 2012), and value based adoption model (Kim et al., 2007), and consumer decision making literature by capturing the asymmetric and symmetric relationships.

Methodologically, the application of the asymmetric approach (*fs*QCA) will disclose how the combinations of technology adoption aspects give equivalent strategies to increase usage behavior. This is a substantial addition to the previous empirical research, which has mostly focused on the net influence of decision-making components (Alam et al., 2020; Awan et al., 2022). In order to better grasp the complexity of combinatorial complications, this technique assumes asymmetric linkages rather than symmetrical effects solely.

Variables causal patterns are examined using complexity and configuration theories to determine how SW purchasing decisions are influenced. According to Woodside (2014), ideas about equifinality (i.e., numerous complex combinations of the same situations can describe the same result) and causal asymmetry (i.e., the reasons for the existence of output are likely to be distinct from the reasons for its absence) are rooted in these theories (Ragin, 2008). As a result, the following research questions are prepared to offer:

**RQ.1** How do numerous elements impact customers’ purchasing decisions for a smartwatch?

**RQ.2** Which variables are essential or sufficient to generate causal configurations that explain how consumers buy a smartwatch?

**RQ.3** What are the possible configurations of factors to decide smartwatch buying for male and female consumers?

## Theoretical Background

### Unified Theory of Acceptance and Use of Technology

Researchers have utilized the Unified Theory of Acceptance and Use of Technology (UTAUT) to examine how new technologies and innovations are adopted (Venkatesh et al., 2003). Researchers used this model to explain the factors identified in this model to buy new technologies and innovative products such as 5G technology (Mustafa et al., 2022), automated public transport (Madigan et al., 2017), users’ home telehealth services (Cimperman et al., 2016; Sohail et al., 2022), etc. UTAUT comprises social, economic, and psychological factors that affect consumers’ decision-making to buy and use a new product. We have picked these factors from UTAUT to understand the smartwatch buying behavior. The bulk of research investigated whether customers’ behavioral intentions to buy new technologies employed a variance-based method. We have combined the concept of *equifinality* with it and explained the different patterns of consumer decision-making.

### Theories of Complexity and Configuration

Despite the complex interactions between variables, many possible combinations explain low and high scores on one measure. The principle of *equifinality* and complexity theory both support the notion that a result may be explained by several causal circumstances (Fiss, 2011; Woodside, 2014). Several elements may be combined to explain the outcome. The previously discussed aspects mentioned above are critical when implementing new technology or innovative products. These factors may combine in various ways to determine whether or not a new product will be purchased. Some or all of these reasons may come into play while deciding whether or not to buy new technology. The presence or absence of certain elements may explain behavioral volatility in decision-making. Thus it’s important to look into that. When it comes to users, elements like psychological importance trumps other considerations like price or social impact. Many aspects go into choosing whether a product will be adopted or rejected, and their diverse combinations may describe it in great detail.

An asymmetrical relationship between cause and effect is provided by configuration theory, which claims that the presence or absence of certain conditions affects an outcome (Fiss, 2011). An asymmetrical relationship might exist between outcome and predictors. No matter how insufficient one variable may be to achieve the goal, it is still necessary for the same result to occur (Fiss, 2011; Woodside, 2014). A required condition is an element that occurs in every configuration and contributes to the elucidation of the result, therefore making it necessary for the outcome. Although the variables identified in UTAUT are vital to making a buying decision, It is undetermined how the presence or absence of these factors affects the rejection or acceptance of technical innovations. Instead of all factors being present in one configuration, the other configuration can contain the present factors but not all. Consequently, the same outcomes may be obtained by varying the presence or absence of some factors combined with others. Hence based on these facts, we propose four below mentioned proposition (Figure 1).

**FIGURE 1:** Conceptualmodel.

#### Proposition 1

A decision to buy a smartwatch isn’t caused by a single ideal combination of social, psychological, and economic elements; rather, several equally effective configurations are available.

#### Proposition 2

Variations in the cause-and-effect relationships might lead to alternative explanations for customer preference for smartwatches purchases.

#### Proposition 3

Smartwatch purchase decision will need the cohabitation of social, psychological, and economic aspects.

#### Proposition 4

Different conditions act differently for male and female consumers. Purchasing decisions and core conditions behind buying differ for both genders, representing the male and female consumer psyche.

### Related Literature

#### Cost Value

Customers are heavily influenced by economic factors when it comes to buying decisions. It’s common knowledge that people purchase or reject products depending on their financial status. According to recent research, consumers’ propensity to buy new products is heavily influenced by the price (Mustafa et al., 2022). The lowest feasible expenses and best possible return on investment are considered part of cost value (Mustafa et al., 2021). The “cost value” is the perceived benefit minus the related expense for a certain product (Venkatesh et al., 2003; Sohail et al., 2021b). The fair choice theorem states that price value finds a balance between costs and profits in operational expenditures (Boudon, 2008).

#### Social Influence

Several technology purchase models look at social aspects as determinants of technology use. The most important social factor in technology acceptance models is social influence. “Social influence” may be defined as someone considering the opinions of others to be substantial enough to buy the product (Venkatesh et al., 2003). The term “social influence” is widely used to describe the impact others have on a person’s choices (Sohail and Delin, 2013; Khan, and Qudrat-Ullah, 2021). Individual viewpoints and societal repercussions have a big role in new product purchases (Mustafa et al., 2022). A study on the utilization of technology-related services revealed that social influence has a significant impact on buying and use behavior of consumers (Mustafa et al., 2022). Another study on consumer use of logistic technology found social influence as a significant factor (Cai et al., 2021).

#### Performance Expectancy

Performance expectancy means the consumer expected value of a system such as a mobile internet technology in carrying out their daily activities (Venkatesh et al., 2003). Perception of performance is a good indicator of future desire to utilize technology or innovative products. Performance expectancy is used in mobile app research to describe behavioral and functional intentions (Chipeva et al., 2018; Sohail et al., 2021a). A study found that perceived performance in mobile phone services was a significant predictor of future satisfaction and use (Mustafa et al., 2022). Researchers found that performance expectancy is a significant factor behind electronic vehicle adoption (Mustafa et al., 2021). Performance expectancy is a significant variable in logistic technology usage (Cai et al., 2021).

#### Effort Expectancy

Effort expectancy (EE) means the system’s or innovative product’s simplicity of use (Venkatesh et al., 2003). Researchers found that EE is a key factor in purchasing any technical product because if the product is easy to use, consumers buy it compared to complex and hard-to-learn products (Cai et al., 2021; Rafique et al., 2021). Mustafa et al. (2022) claim that when new technology is readily accessible and easy to use, people are more receptive. The same findings were revealed in the buying decision of electric vehicles if they are easy to use and operate; consumer wants to buy them (Sohail et al., 2013; Mustafa et al., 2021).

#### Facilitating Conditions

Facilitating conditions (FC) is a term that refers to the tools and resources used to take advantage of technology or innovative product (Venkatesh et al., 2003). Like in this study, smartwatches are associated with smartphones and the internet. If a consumer does not have a smartphone or the internet, a smartwatch is less effective. Several researchers found that facilitating conditions are positively associated with the buying decision of consumers in technical and innovative products such as mobile internet (Venkatesh et al., 2003), mHealth adoption (Alam et al., 2020), usage of logistic technologies (Cai et al., 2021), electronic vehicles purchase (Mustafa et al., 2021), 5G adoption (Mustafa et al., 2022) etc.

#### Gender and Buying Behavior

Researchers (Schindler and Holbrook, 2003) discover that males exhibit sentimental attachment to the styles they encountered in their childhood, while women do not—that is, their preferences peaked for fashionable things during their youth. In another study, researchers revealed that for women, promotional gifts have a greater influence on their future purchasing habits (vs. men). As a result, women are more motivated to reciprocate since they get more transactional value from a promotional purchase than men (Alroobaea et al., 2020; Kovacheva et al., 2021). For female customers, a soft hand movement is preferred over a fast one since it makes the product and the action performer seem more feminine to the audience (Malik and Sayin, 2022). Both men and women similarly received textual information, but men were more inclined to depend on the product’s color to determine its healthiness (Meng and Chan, 2022). This literature concluded that gender does matter in consumers’ purchase decisions. Hence, we have applied the configuration and complexity approach to identify the different unique configurations to understand the buying patterns of male and female consumers.

## Methodology

### Fuzzy Set Qualitative Comparative Analysis

Fuzzy-set qualitative comparative analysis combines fuzzy sets with logic principles in Qualitative Comparative Analysis (Ragin, 2008). The *fs*QCA has been used in technology adoption (Mustafa et al., 2022), knowledge management (Sahibzada et al., 2020b), strategy and organizational research (Fiss, 2011), organizational performance (Farooq Sahibzada et al., 2021) and so on.

The *fs*QCA method is a case-based strategy that emphasizes the interaction between variables. Various processes or variables are assumed to be autonomous and interdependent in this model. The core assumption is that there are a plethora of solutions or paths that may get to the same result. The same elements may have various effects in this technique, but different circumstances may be necessary or sufficient to achieve a certain result (Rihoux and Ragin, 2008; Woodside, 2014). *fs*QCA is useful for developing, elaborating, and testing hypotheses, both inductively and deductively (Mustafa et al., 2022). It is also helpful to look for particular instances in the sample; *fs*QCA can help locate and investigate various conditions that might explain the high scores received for the same result (Pappas and Woodside, 2021).

On the contrary, variance-based (v-b) analysis reveals a single ideal solution, limiting the possible options (Woodside, 2013). When *fs*QCA is used instead of typical analytical methods, it is possible to get many benefits. Qualitative and quantitative assessments are combined in *fs*QCA, and it calculates how much a case belongs to a set (Rihoux and Ragin, 2008). It does this by connecting the qualitative and quantitative domains. Simpler models and a less rigorous methodology are used in v-b techniques to evaluate variables.

Meanwhile, *fs*QCA digs deeper and explains complex and asymmetric relations (Pappas and Woodside, 2021). Instead of employing typical v-b procedures, *fs*QCA uses various configurations of explanatory factors that include variables not found through more classic methods (Woodside, 2014). Because the sample is divided into subsets using *fs*QCA, numerous conditions may be examined simultaneously. Some possible solutions will have an outlier, but not all will (Pappas and Woodside, 2021). Because the v-b technique is impervious to outliers, *fs*QCA has a higher level of resilience than v-b approaches (Fiss, 2011).

There are several configurations (or solutions) in *fs*QCA that may have necessary variables present or negated in a solution (i.e., not present). As a result, they may not be a part of the solution since they don’t immediately influence a solution. Both “core” and “peripheral” factors may be present (or absent) to show a strong or weak causal relationship between the outcome and precursors (Fiss, 2011).

### Research Context

Given our study’s goal, we selected China as our test location. China is the most populated country globally, making it the world’s most important market for any new technology. We received replies from Chinese residents and foreigners residing in China for employment, business, or research to guarantee that our study’s conclusions are consistent and accurate. Additionally, we sent out questionnaires to all major cities to get the most diverse data (Beijing, Shanghai, Guangzhou, Shenzhen, Wuhan, and Tianjin).

### Instrument Design and Data Collection

We used a construct that has already been tested and proven effective. Appendix A1 describes how each measurement item is set out and its specifications. We adjusted the original construct according to our study goal by slightly changing the wording to be more helpful. We have translated the original construct according to the requirements of our sample population. Academicians were consulted for this purpose. Questionnaire star Chinese^4^, an online platform, was used for survey and data collection because it is a robust way to collect data and avoid manual data entry. We have conducted an online survey for 9 weeks to collect valid 468 responses (Alroobaea and Mayhew, 2014). Seven hundred twenty questionnaires were distributed and completed 468 responses were received with a response rate of 65%, which explains our survey’s success because researchers explain if the response rate is above 50%, a survey is considered successful and collected the required information to carry on a study (Lindemann, 2021). We have distributed Table 1 presents the demographic characteristics of our sample. We have used a seven-point Likert scale to record the consumers’ responses, where 1 indicates strongly disagree to 7 strongly agree.

**TABLE 1:** Demographic profile of the respondents.

		Frequency	Percent
Gender	Male	268	57.26%
	Female	200	42.73%
Age	18–25 years	114	24.35%
	26–35 years	172	36.75%
	36–45 years	125	26.70%
	>45 years	57	12.17%
Education	High School	19	4.05%
	Bachelor	173	36.96%
	Master	270	57.69%
	Doctorate	6	0.01%
Occupation	Student	1	0.002%
	Govt. Employee	130	27.77%
	Private Company Employee	190	40.59%
	Businessman/women/other	147	31.41%
Residential Status	Chinese	324	69.23%
	Expatriate	144	30.76%
	Total	468	100.00%

### Common Method Bias

A common method bias might exist when the same respondent provided data for both the predictor and the outcome variables, then analyzed using the same instrument. We estimated CMB following the approved procedural and statistical procedures (Hew et al., 2019; Masud et al., 2021). Throughout the data gathering process, we maintained the anonymity of our respondents and made it clear that there was no right or wrong answer. We have mentioned at the start of our questionnaire that this study is only for academic purposes, and information provided by consumers will remain confidential regarding their personal information. Participants were requested to add their cell numbers to avoid duplicate attempts.

Apart from the statistical measures, Harman’s single factor test was used to determine whether a single component accounts for most of the covariance across all constructs. The data showed that the first component only accounted for 35.34 percent of the overall variance, much lower than the conservative threshold of 40% (Hair et al., 2014). This study’s findings proved that the typical technique bias was not a major issue.

### Reliability and Convergent Validity

First of all, we have checked the collinearity in the dataset. According to experts, data has no collinearity issues if the VIF values are less than 5 (Hair et al., 2014). The results of the present investigation showed the inner VIF values are lower than the cutoff point (between 1.384 and 2.972). It shows that the data utilized in this study are not collinear (Table 2). Furthermore, Indicator reliability and convergent and discriminant validity of the model’s construction should be used to establish an evaluation of the measurement model (Hair et al., 2014). Reliability was assessed using Cronbach’s Alpha (α) and indicator loading calculations. Convergent validity was evaluated on the construct indicator to see whether it appropriately assessed the research variables. AVE measures the total variation in the indicators used to compensate for the latent construct.

**TABLE 2:** Reliability and validity analysis.

Constructs	Items	Loadings	T-values	VIF	α	CR	AVE
Cost Value	CV1	0.792	29.256	1.421	0.719	0.842	0.639
	CV2	0.798	29.107	1.422			
	CV3	0.809	39.103	1.384			
Effort Expectancy	EE1	0.864	30.628	2.555	0.874	0.914	0.726
	EE2	0.881	33.183	2.761			
	EE3	0.86	23.888	2.358			
	EE4	0.803	18.990	1.898			
Facilitating conditions	FC1	0.829	42.566	2.111	0.877	0.915	0.730
	FC2	0.849	50.384	2.349			
	FC3	0.866	49.161	2.607			
	FC4	0.873	56.484	2.385			
Performance Expectancy	PE1	0.876	57.358	2.673	0.909	0.936	0.786
	PE2	0.892	68.218	2.867			
	PE3	0.888	66.473	2.778			
	PE4	0.889	72.250	2.768			
Social Influence	SI1	0.898	65.095	2.972	0.895	0.927	0.760
	SI2	0.893	78.882	2.874			
	SI3	0.873	57.699	2.624			
	SI4	0.822	35.577	2.185			
Use Behavior	UB1	0.877	51.689	2.113	0.849	0.909	0.768
	UB2	0.871	48.568	2.036			
	UB3	0.882	67.738	2.049			

In contrast, CR is a measure of the consistency of the variables. Items’ reliability is shown in Table 2, where factor loadings on key structures influence the item’s reliability. A factor loading of at least 0.6 was required for a component to be considered significant and included in the model (Hair et al., 2014). It is also important to note that Cronbach’s alpha for all constructions is more than or equivalent to 0.7, which is acceptable (see Table 2).

The study has also looked at how reliable the constructs are when measured using composite reliability rather than Cronbach’s alpha, a comparatively better approach (Werts et al., 1974). Variables are more reliable when the composite reliability value for the construct is greater than 0.07. Convergent validity was established when all constructs’ average extracted variance (AVE) estimations exceeded 0.50 (Hair et al., 2014; see Table 2).

### Discriminant Validity

The Fornell-Larcker criteria are used to assess the discriminant validity of the proposed model. According to Table 3, discriminant validity is proven using the Fornell-Larcker criterion since the top value of each column’s association of measures is maximal (Hair et al., 2014).

**TABLE 3:** Fornell-Larcker criterion.

	Mean	Std	CV	EE	FC	PE	SI	UB
CV	4.659	1.755	0.800					
EE	4.306	1.156	0.018	0.852				
FC	5.208	1.422	0.402	0.157	0.854			
PE	4.736	1.599	0.594	0.213	0.552	0.886		
SI	4.927	1.584	0.693	0.253	0.586	0.807	0.872	
UB	4.669	1.638	0.565	0.192	0.544	0.771	0.775	0.877

*Gray values represent the validity of results, compared to other values presented in the table. Diagonal values should be greater than others.*

Henseler et al. (2015) suggested a unique approach for discriminant validity determination. They argued that although the Fornell-Larcker criteria measure discriminant validity successfully, it cannot detect its absence.

As a consequence, the discriminant validity of HTMT was found. Table 4 contains the HTMT values for the variables utilized in this investigation. According to the requirements, the HTMT values of all variables must be less than 0.90 (Hair, J. F. et al., 2016; Bari et al., 2019). The table below shows that all measures had HTMT values less than 0.90, suggesting that all variables under examination exhibit discriminant validity.

**TABLE 4:** HTMT ratio.

	CV	EE	FC	PE	SI	UB
CV						
EE	0.063					
FC	0.507	0.181				
PE	0.736	0.239	0.617			
SI	0.869	0.287	0.662	0.806		
UB	0.721	0.223	0.627	0.817	0.825	

### Contrarian Case Analysis

We conducted contrarian case analysis before implementing *fs*QCA in accordance with (Woodside, 2014; Pappas and Woodside, 2021). It enables a straightforward and rapid examination of the proportion of occurrences in our sample that are unaccounted for by main effects and hence excluded from a normal variance-based technique (Woodside, 2014). We evaluate whether one variable has a positive or negative influence on another based on the assumption that most observations in a sample corroborate this connection. However, a portion of the sample’s examples may demonstrate the opposite relationship. Contrarian examples do arise independently of the degree of the primary effects; consequently, the occurrence of contrarian cases may be investigated by a contrarian case study (Woodside, 2014).

The sample is divided into quintiles. Avoid doing median splits on continuous variables to limit statistical power and the possibility of erroneous findings (Fitzsimons, 2008). Following that, we used cross-tabulations to determine the degrees of linkage between the quintiles. The upper left and lower right instances illustrate primary impacts, whereas the bottom left and top right cases illustrate secondary effects (Appendix A2). These are instances that are outliers in our dataset. The data reveal that numerous factors interact independently of the principal impact, emphasizing the significance of doing a configurational analysis.

### Fuzzy Set Qualitative Comparative Analysis

#### Calibration

In order to employ the *fs*QCA technique, the raw data must be transformed into fuzzy sets with values ranging from zero (complete omission from a set) to one (complete inclusion) (Ragin, 2009). An index is created for each construct by averaging its related indications before calibrating the variables. Three anchors are required during the calibration process: full membership, full non-membership, and a crossover point. In this work, theoretical anchors created by early researchers are used to calibrate fuzzy sets (Sahibzada et al., 2020a; Mustafa et al., 2022). Since this research employed seven-point Likert scales, we selected these cutoff points: 6 for full set membership, 4 for crossover, and 2 for full set non-membership by following (Mustafa et al., 2022). We used fsQCA version 3.1 to calibrate the data in our investigation. *fs*QCA excludes situations that are exactly 0.5 from the research, making it harder to investigate circumstances that are precisely 0.5 (Being a part of a certain group; Ragin, 2009; Sahibzada et al., 2022). Fiss (2011) suggests adding a constant of 0.001 to the causal conditions below complete membership scores of 1 to remedy this problem. Following the advice of Fiss, we’ve added an extra 0.001 constant to our code to be sure this doesn’t happen.

#### Analysis of Necessary Conditions

Fuzzy set qualitative comparative analysis next step is to generate a truth table, but first, we check to see whether any causal conditions are required. There is a consistent interpretation given to the results of the *fs*QCA research. When the value of consistency exceeds 0.9, the condition becomes essential (Mustafa et al., 2022). This condition analysis’s findings are shown in Table 5. For the implementation of buying behavior of SW, we examined the prerequisites. The findings showed that facilitating conditions, performance expectancy, and social influence were necessary for a decision.

**TABLE 5:** Necessity analysis (overall sample).

Condition tested	Consistency	Coverage
*EE*	*0.722*	*0.801*
∼EE	*0.472*	*0.765*
*FC*	***0.930***	*0.789*
∼FC	*0.212*	*0.625*
CV	*0.846*	*0.848*
∼CV	*0.325*	*0.626*
*PE*	***0.913***	*0.889*
∼PE	*0.269*	*0.548*
*SI*	***0.940***	*0.860*
∼SI	*0.225*	*0.531*

*The symbol ∼ denotes the absence of the condition. The bold values represent the conditions that are necessary for an event/outcome, the final concluding value results after the necessary test.*

#### Obtaining the Fuzzy Set Qualitative Comparative Analysis Solutions

The “*fs*QCA method outputs a truth table with 2*^k^* rows, where “k” is the number of result predictors” once the calibration and analysis of necessary conditions are finished. Each column in the table offers a potential combination. We chose 4 as the frequency cutoff and 85% as the consistency cutoff points to achieve viable solutions by following (Fiss, 2011; Pappas and Woodside, 2021). “Frequency” refers to the total number of observations taken for each conceivable combination. A solution’s consistency may be defined as “the degree to which cases conform to the set-theoretic connections represented in the solution.” In order to acquire enough empirical data to investigate subgroup relations, researchers advise setting a cutoff frequency. Larger samples (e.g., 150 or more cases) should have a larger cutoff value than small and medium samples (Ragin, 2009). A complex solution, a parsimonious solution, and an intermediate solution were obtained using the Quine–McCluskey approach when cutoff points were used. We followed Fiss in result interpretation; he claims that a more complete and aggregated picture of the outcomes may be obtained by combining the parsimonious and intermediate solutions (Fiss, 2011).

Additionally, these solutions are validated by essential and sufficient core and peripheral requirements. “Core” conditions or elements, i.e., critical components, cannot be excluded from any configuration (i.e., variables with a strong causal relationship to the outcome) and are often found in intermediate and parsimonious solutions. In comparison, “peripheral” conditions are less crucial and may even be interchangeable (i.e., elements with a weak causal connection to the result). They are often found exclusively in intermediate solutions (Mustafa et al., 2022). These criteria may or may not be present in a solution, or they may be irrelevant (i.e., “do not care”) (Fiss, 2011). In a “do not care” situation, conditions may exist or not exist.

To facilitate comprehension of the findings, we defined and described each arrangement’s core and peripheral circumstances, as recommended by Pappas and Woodside (2021). To demonstrate, black circles (•) and crossed-out circles (⊗) denote the existence and absence of an item, respectively. Large circles represent core circumstances, small circles represent peripheral conditions, and blank regions represent a “do not care” state. The solution’s total consistency score of 0.936, as shown in Table 6, indicates that the causal combination secures the result. The results indicated that the entire solution gave a sufficient degree of coverage 86.5%, with 86.5% of instances exhibiting buying configurations for SWs by these six configurations. Similarly, all identified configurations had a high degree of consistency (more than the 0.75 criteria) and coverage, indicating that the model was informative (Woodside, 2013). The total solution coverage metric represents the degree to which SW buying decision can be predicted given a collection of configurations and is comparable to the correlational *R*-square value.

**TABLE 6:** Configurations for buying smartwatches.

	Solutions to buy a smartwatch					

Configurations	1	2	3	4	5	6
CV	🌑	⊗			🌑	🌑
PE		🌑	🌑		🌑	🌑
SI			🌑	🌑	🌑	
FC			•	•		•
EE	⊗	•		•		
Consistency	0.888	0.897	0.925	0.903	0.932	0.935
Raw coverage	0.435	0.268	0.846	0.668	0.786	0.764
Unique Coverage	0.010	0.008	0.022	0.020	0.019	0.005

*Overall solution consistency*	**0.865**					

*Overall solution coverage*	**0.936**					

*Black circles (🌑) indicates the presence of a condition, and circle with “x” (⊗) indicates its absence, while blank space indicates “don’t care condition.” Large circle: core condition, small circle: Peripheral condition. PE, performance expectancy; CV, cost value; EE, effort expectancy; SI, social influence; FC, facilitating conditions.*

Truth table results revealed that Cost value, Performance expectancy, and Social influence in buying Smartwatches are the core(key) conditions. In contrast, effort expectancy and facilitating conditions are peripheral conditions (have a weak causal relationship with the outcome). Solution 1 contains Cost value as a core condition and the absence of Effort expectancy. At the same time, the rest of the variables are not present in this solution, which means consumers do not care about the rest of the variables while making a decision. In solution 2, with the absence of a cost factor, PE is a key factor with EE as a secondary level factor. Solution 3 and 6 represent two core factors with one secondary factor, i.e., FC. In solution 3, PE and SI, whereas in solution 6, Cost and PE are key factors behind decision making. Solution 4 contains SI as a key factor, with FC and EE as peripheral factors. Solution 5 combines all three core factors behind decision-making, i.e., CV, PE, SI (Table 6).

Furthermore, we have followed the procedures mentioned above to produce exclusive solutions for male and female users. Necessity analysis test for female consumers revealed that social influence and facilitating conditions are necessary, whereas perceived expectancy along with these two conditions are necessary for male consumers (Table 7). Truth table results based on gender are presented in Table 7. Results revealed that social influence is a core condition for female consumers, whereas social influence and perceived expectancy are core conditions for male consumers. Consistency of individual and overall solutions identified for both gender are well above the threshold value of 0.75 (Woodside, 2013). Overall solution coverage for male and female consumers is also considerably high, as it explains 87.7% buying pattern for females and 91.4% for male consumers with a high consistency of 0.875 and 0.900, respectively (Table 8).

**TABLE 7:** Necessity analysis.

	Female		Male	
	
Condition tested	Consistency	Coverage	Consistency	Coverage
EE	*0.7257*	*0.7871*	*0.7195*	*0.8123*
∼EE	*0.4779*	*0.7728*	*0.4679*	*0.7603*
FC	***0.9226***	*0.7681*	***0.9357***	*0.8065*
∼FC	*0.2288*	*0.6746*	*0.2010*	*0.5896*
CV	*0.8407*	*0.8406*	*0.8509*	*0.8540*
∼CV	*0.3382*	*0.6261*	*0.3164*	*0.6268*
PE	*0.8928*	*0.8876*	***0.9285***	*0.8913*
∼PE	*0.3056*	*0.5718*	*0.2427*	*0.5282*
SI	***0.9280***	*0.8521*	***0.9499***	*0.8661*
∼SI	*0.2537*	*0.5622*	*0.2048*	*0.5064*

*The symbol ∼ denotes the absence of the condition. The bold values represent the overall consistency and coverage of results, different from individual results crux of the findings.*

**TABLE 8:** Gender-specific solutions to buy smartwatches.

	Buying solutions for female			Buying solutions for male				
	
Configurations	1	2	3	1	2	3	4	5
CV	•		•	⊗				•
PE			•	🌑	🌑	🌑	🌑	
SI	🌑	🌑	🌑		🌑	🌑		🌑
FC	•	•			•		•	•
EE		•	•	•		•	•	•
Consistency	0.893	0.889	0.940	0.895	0.932	0.930	0.929	0.928
Raw coverage	0.778	0.653	0.572	0.268	0.860	0.671	0.664	0.606
Unique coverage	0.204	0.079	0.019	0.006	0.206	0.009	0.005	0.022

*Overall solution consistency*	**0.875**			**0.900**				

*Overall solution coverage*	**0.877**			**0.914**				

*Black circles (🌑) indicates the presence of a condition, and circle with “x” (⊗) indicates its absence, while blank space indicates “don’t care condition.” Large circle: core condition, small circle: Peripheral condition. PE, performance expectancy; CV, cost value; EE, effort expectancy; SI, social influence; FC, facilitating conditions.*

#### Predictive Validity

Predictive validity validation of our solutions is critical. The model’s predictive validity has been established if the explained variable can be reliably predicted in multiple samples (Woodside, 2014). According to previous researchers’ instructions (Pappas and Woodside, 2021; Mustafa et al., 2022), we divided our sample into holdout samples and subsamples for this reason (234 observations for each). The holdout dataset was used to calculate a new solution 1 variable in the second phase. Our analysis and cutoff points are identical to those used on the complete sample. Table 6 displays the results of the subsample’s solutions. In the “XY Plot” (Figure 2), we can see how solution 1 compares to the “XY Plot.” For smartwatch purchase, Solution 1 gave us coverage of 0.815 with a consistency of 0.930, whereas the “XY Plot” shows the consistent findings, 0.878 coverage with a consistency of 0.921. These calculations show that the data are largely consistent at 89.8%, and these five solutions are a subset of consumer decision-making to buy smartwatches, and their coverage is 89.3% (Table 9). We have shown that the high consistency subsample models can reliably predict the holdout samples and vice versa for all models in our predictive tests (Figure 2).

**FIGURE 2:** Models 1 and 2 are tested using data from the holdout sample.

**TABLE 9:** Solutions from the subsample.

	Models from subsamples	Raw coverage	Unique coverage	Consistency
S1	FC*PE*SI	0.815	0.026	0.930
S2	SI*CV*FC	0.768	0.018	0.918
S3	SI*FC*EE	0.628	0.010	0.911
S4	SI*PE*EE*CV	0.550	0.016	0.943
S5	PE*CV*EE*FC	0.544	0.009	0.949

Overall solution coverage: 0.893. Overall solution consistency: 0.898. * Represents the combined effect of presented conditions in each row, e.g., S1–S5.

## Discussion

This research aims to provide a comprehensive and integrated evaluation of consumers’ decision-making processes regarding the purchase of smartwatches and understand gender differences in a purchase decision. These conclusions are based on the relevant literature and complexity theory to comprehend how various combinations of psychological, economic, and societal elements lead to conditions favorable to the widespread purchase of SW and consumers’ purchasing psyche. According to our *fs*QCA results, three of these elements are necessary for decision-making (RQ.2). Alternatively, six combinations are causally sufficient configurations for the whole sample to enhance consumers’ proclivity to purchase SW, elucidating the phenomenon’s complexity (RQ.3). While facilitating conditions, performance expectancy, and social influence are core conditions (Primary considerations), cost value and effort expectancy are peripheral or secondary level variables in buying SWs. No single sufficient factor motivates consumers to buy SW (RQ.2). Results proved that consumer decision-making is a complicated process, and different factors influence consumer decision-making in different capacities and strengths to make a decision.

Solution 1 consists of cost factor (core condition) and absence of effort expectancy. It reflects the decision preferences of those users who are more concerned about the economic factor, and effort expectancy does not play any role in their decision-making. In contrast, they do not much care about the rest of the variables, i.e., the presence or absence of these factors does not affect their decision-making approach. In short, this segment of users only considers cost factors before deciding. These findings are consistent with scholars who claim that economic factors play a key role in making buying decisions (Dhiman et al., 2019; Mustafa et al., 2022).

Solution 2 contains the PE as the core condition (key factor) with the absence of cost value and EE as a secondary level factor to decide. Users in this solution care about their psychological perception of the smartwatch and do not consider economic factors when deciding to buy. In line with the studies claim that psychological factors are important for decision making (Cai et al., 2021; Mustafa et al., 2022).

Solution 3 contains SI and PE as key factors behind decision-making along with the FC as a peripheral condition. It means users under this solution pay more attention to the expected performance of SW, and their decisions are influenced by their social circle. According to solution 4, a set of consumers decide after considering their social circle with a little consideration of FC and EE. It means a user who has a smartphone, and it’s easy for them to learn how to use SW consider with their fellows, and it convinces them they buy SWs. These solutions are consistent with the findings of Alam et al. (2020) and Mustafa et al. (2022), who claim that social influence plays a key role in technology adoption.

Solution 5 provides information about those users who follow the three key factors to make their buying decision, i.e., they think about the cost factor, PE, and consider their social circle before making a purchase decision. At the same time, the sixth solution provides information about those users’ decision-making preferences who do not pay much importance to their social circle. They compare cost factors with performance expectancy, consider facilitating conditions at secondary level factors and decide their buying (Venkatesh et al., 2012; Mustafa et al., 2021).

For female consumers, social influence emerged as a core condition means female consumers consider their circle of friends or family before buying a product and are highly influenced by their social circle. Solution 1 for female consumers identifies that a segment of female users pays more attention to the product’s price and its facilitating conditions and social influence before making a final decision. At the same time, female consumers who follow the second solution are more concerned about effort expectancy than price with SI and FC. Female consumers who follow the third solution to make buying decisions consider all understudy factors except FC. The third segment of female consumers is more conscious and thinks more than the other two segments before purchasing.

Fuzzy set qualitative comparative analysis results divide the male portion of our sample into five segments and explain their characteristics of buying behavior. Performance expectancy and social influence are revealed as core conditions for male consumers. Male consumers who follow solution 1 to decide to buy a product do not consider price factors and emphasize performance expectancy and effort expectancy of a product. It means these male consumers are quality conscious and do not compromise on the perceived performance. Male users segments two and three behave almost identical. They follow solutions 2 and 3 to decide before buying a product. They are more concerned about performance expectancy and social influence with facilitating condition (s2) or effort expectancy (s3). We can say these are those users who are well aware of the new product market but highly influenced by their social circle, i.e., if someone from their social circle buys a new phone or new SW, they will start considering buying it. Segment four of male users do not pay more importance to price or social opinion and go for those products that fascinate them. They carefully consider PE, FC, and EE before their buying decision. The fifth segment of male users is the most conscious among male consumers as they consider every possible factor before buying a product.

In a nutshell, if we compare buying behavior of male and female users following important facts have been revealed in this study (P4).

1. Male consumers are more quality conscious, whereas females are more socially influenced in their buying decisions.
2. Females are more price-conscious than their counterparts.
3. Not all, but few consumers behave almost identical regardless of gender (S3 For females, S5 for males).

### Theoretical Implication

The theoretical significance of this work emerges from its novel approach and technique. Our technique is distinct from most research that has examined consumers’ decision-making preferences using variance-based methodologies, for example (Alam et al., 2020; Gul et al., 2021; Awan et al., 2022; Jamil et al., 2022). These techniques assume the symmetrical relationship between variables, which may not accurately reflect actual occurrences owing to the potential of asymmetric interactions between variables (Fiss, 2011; Woodside, 2017; Mustafa et al., 2022). The asymmetric relationship between users’ performance expectancy, social influence, cost, effort expectancy, and facilitating conditions is better represented by utilizing fsQCA based on complexity and configuration theories. It results in the generation of new ideas and theories.

In most previous studies, gender is treated as a control variable (Mustafa et al., 2022), exploratory variable (Malaquias and Hwang, 2019) or moderator (Venkatesh et al., 2012). We made it a base and studied it as a key factor, as researchers (Malaquias and Hwang, 2019) identified that gender plays a significant role in buying decisions. We have identified different configurations to understand the decision-making of male and female consumers. Furthermore, we have compared the preferences of consumers based on gender and highlighted different characteristics of male and female consumer psyche.

Additionally, we contribute to and enhance previous research using fsQCA (Venkatesh et al., 2003; Alam et al., 2020; Mustafa et al., 2021), etc., by developing precise propositions that enable us to distinguish distinct categories of users in our sample; we also contribute to the theory development. The configurations illustrate how multiple individuals with similar motivations, emotions, sentiments, and needs exhibit varying decision-making capacities. The findings demonstrate complicated relationships between the variables affecting buying decisions and the asymmetric interactions that result in the same outcome. The empirical findings show that users with comparable levels of motivation and emotion do not equally perceive products and will have diverse preferences to buy. Additionally, we examine our model’s predictive validity using subsamples, a technique that is not as often used in empirical research as model fit testing (Pappas and Woodside, 2021; Mustafa et al., 2022). Model fit testing alone is insufficient since even a well-fit model may fail to predict the outcome properly (Pappas and Woodside, 2021).

Distinct from previous research that utilized variance-based methodologies to evaluate if a variable is substantial or not for a result. We significantly clarify and explain the complication of the decision-making procedure that certain aspects may not contribute as major or core conditions in consumer decision-making. Still, they may play a minor part in creating a persuasive judgment. It is the more reasonable explanation of possible variables underlying decision-making.

Our research is one of the first to combine configuration and complexity theories with *fs*QCA in order to provide necessary and sufficient criteria for elucidating consumers’ decision-making preferences. Prior research has found many antecedents to buying products, including performance expectancy, cost value, effort expectancy, social influence, facilitating conditions (Venkatesh et al., 2003). Our results, however, reveal that depending on their combination, these characteristics may represent a core, peripheral, or no association with decision-making and, therefore, that no one-size-fits-all solution exists. The study results expand the canvas of complexity and configurational theory in terms of consumer decision-making to buy innovative products.

This study adds to existing research on technology adoption by providing a new viewpoint on how many factors interact to explain consumers’ preferences to buy new products. The previous study has shown a direct correlation between PE, EE, SI, CV, FC, and innovative product use (Venkatesh et al., 2003). Numerous combinations discovered in this research show that multiple configurations should be employed when examining user feelings, preferences, and satisfaction with new products. There is a better possibility that identified configurations explain the behavior of consumers in the sample and the behavior in general. Thus, we demonstrate the link between various degrees of perceptions, desires, and emotions and their influence on accepting new products (smartwatch). Generally, this relationship has received less attention in the past. Lastly, its worth mentioning that consumers’ decision-making in buying smartwatches has never been extensively investigated. We have uncovered the complexity of smartwatch users’ buying decisions by conducting this study.

### Practical Implications

This research provides scientific evidence to help SW producing firms, advertising agencies, and key decision-makers. Six unique configurations of psychological, social, and economic factors may be employed to increase SW sales and better understand customer behavior. Smartwatch producers may choose from various alternative solutions for achieving their goals, considering each SW market’s cultural, social, and economic features. Smartwatch producing companies can also improve their features after examining consumer preferences. For example, reducing the price will surely give them a competitive advantage as consumers in developing countries are especially price-conscious. As the characteristics mentioned above of every market differentiae with geographical boundaries, emerging and small smartwatch producing companies can target developing countries.

## Limitations and Recommendations

While we made every effort to include all relevant components of our research, it is limited in various ways. Firstly, we drew our sample from a single country. Consequently, psychological, cultural, economic, and social characteristics may vary significantly among regions. As a consequence, we advocate conducting the same survey across more geographic boundaries to have a better understanding of user decision-making. Second, we did not collect data on our target population’s income level, which might affect consumers’ decision-making choices. Thus, future research should gather data on the target population’s income level and study its influence on SW users’ decision-making preferences. Thirdly, *fs*QCA does not keep track of each factor’s unique contribution to each solution; rather, *fs*QCA identifies complicated combinations of factors and the percentage of the result explained by these configurations. Additionally, we did not separate the male and female users’ preferences or check the decision-making function in different age groups. Further studies can work on these aspects. Lastly, we recommend the *fs*QCA approach to understand consumers’ technology adoption and behavior fluctuation across different industries because it explains the variables’ relationship and their impact on output better than multivariate models.

## Data Availability Statement

The datasets presented in this study can be found in online repositories. The names of the repository/repositories and accession number(s) can be found below: https://drive.google.com/file/d/1dexlqtfS8RR_64IXppYv4oHsAANvcY1e/view?usp=sharing.

## Author Contributions

SM: conceptualization, methodology, software, and writing – original draft. MS: approved the final draft and data collection. RA and SR: editing, investigation, and data collection. AA and AO: visualization and investigation. MN: review the draft, editing, and handle data flow. All authors contributed to the article and approved the submitted version.

## Conflict of Interest

The authors declare that the research was conducted in the absence of any commercial or financial relationships that could be construed as a potential conflict of interest.

## Publisher’s Note

All claims expressed in this article are solely those of the authors and do not necessarily represent those of their affiliated organizations, or those of the publisher, the editors and the reviewers. Any product that may be evaluated in this article, or claim that may be made by its manufacturer, is not guaranteed or endorsed by the publisher.

## Footnotes

1 Global smartwatch shipment forecast 2025 | Statista.

2 Business News: U.S. Smartwatch Sales Are Soaring - HODINKEE.

3 Global Smartwatch Market Size, Share, Trends & Growth Analysis Report | 2021 to 2026 | COVID-19 impact (marketdataforecast.com).

4
www.wjx.cn

## Appendix

**TABLE A1:** Measurement items.

Variables	Measurement Items		References
Cost Value	*CV1*	The Smartwatch price is reasonable.	Venkatesh et al., 2012; Mustafa et al., 2021
	*CV2*	The price I pay for a smartwatch is well-matched in its value.	
	*CV3*	At the present cost, the smartwatch delivers a good value.	
Effort Expectancy	EE1	Learning how to use smartwatches is easy for me.	Venkatesh et al., 2003; Mustafa et al., 2022
	EE2	It would be easy for me to become skillful at using the smartwatch.	
	EE3	It is clear and understandable to interact with smartwatches.	
	EE4	I would find the smartwatch easy to use.	
Facilitating conditions	FC1	I have the resources necessary to use smartwatches.	Venkatesh et al., 2003; Mustafa et al., 2022
	FC2	I can get help from a service provider when I have difficulties using a smartwatch.	
	FC3	I will use a smartwatch if I have a compatible device.	
	FC4	Smartwatch is compatible with the devices I use.	
Performance Expectancy	PE1	Using the smartwatch increases my productivity	Venkatesh et al., 2003; Mustafa et al., 2021
	PE2	Using the smartwatch enables me to accomplish tasks more quickly.	
	PE3	I find that the smartwatch is useful in my daily life	
	PE4	Using a smartwatch increases my chances of achieving things important to me.	
Social Influence	SI1	Society members who are influential to me think that I must use a smartwatch.	Venkatesh et al., 2003; Mustafa et al., 2022
	SI2	Society members who influence my behavior think that I must use a smartwatch.	
	SI3	Society members whose opinions I value prefer that I use a smartwatch.	
	SI4	I am inspired by society members who use the smartwatch.	
Use Behavior	UB1	I will use a smartwatch in the future.	Venkatesh et al., 2003; Mustafa et al., 2022
	UB2	I will recommend the smartwatch to others.	
	UB3	Smartwatches increase my willingness to use them.	

## Appendix

**TABLE A2:** Contrarian case analysis.

Smartwatch buying decision (UB)													

		1	2	3	4	5			1	2	3	4	5
**EE. (phi^2^ = 0.055, *p* < 0.040)**	**1**	***26(5.56%)***	***16(3.42%)***	**16(3.42%)**	**14(2.99%)**	**22(4.70%)**	**FC. (phi^2^ = 0.418, *p* < 0.001)**	**1**	***43(9.19%)***	***28(5.98%)***	**6(1.28%)**	**3(0.64%)**	**2(0.43%)**
	**2**	***23(4.91%)***	***23(4.91%)***	**14(2.99%)**	**21(4.99%)**	**16(3.42%)**		**2**	***19(4.06%)***	***26(5.56%)***	**24(5.13%)**	**14(2.99%)**	**11(2.35%)**
	**3**	**13(2.78%)**	**18(3.85%)**	**19(4.06%)**	**17(3.63%)**	**20(4.27%)**		**3**	**18(3.85%)**	**17(3.63%)**	**34(7.26%)**	**43(9.19%)**	**17(3.63%)**
	**4**	**22(4.70%)**	**22(4.70%)**	**32(6.84%)**	***38(8.12%)***	***27(5.77%)***		**4**	**5(1.07%)**	**13(2.78%)**	**9(1.92%)**	***21(4.49%)***	***28(5.95%)***
	**5**	**4(0.85%)**	**10(2.14%)**	**9(1.92%)**	***8(1.71%)***	***18(3.85%)***		**5**	**3(0.64%)**	**5(1.07%)**	**17(3.63%)**	***17(3.63%)***	***45(9.62%)***
**CV. (phi^2^ = 0.427, *p* < 0.001)**	**1**	***51(10.9%)***	***19(4.06%)***	**13(2.78%)**	**9(1.92%)**	**9(1.92%)**	**PE. (phi^2^ = 1.048, *p* < 0.001)**	**1**	***62(13.25%)***	***15(3.21%)***	**4(0.85%)**	**3(0.64%)**	**2(0.43%)**
	**2**	***13(2.78%)***	***35(7.48%)***	**10(2.14%)**	**12(2.56%)**	**14(2.99%)**		**2**	***18(3.85%)***	***49(10.47%)***	**19(4.06%)**	**5(1.07%)**	**7(1.50%)**
	**3**	**13(2.78%)**	**13(2.78%)**	**31(6.62%)**	**18(3.85%)**	**14(2.99%)**		**3**	**5(1.07%)**	**11(2.35%)**	**49(10.47%)**	**24(5.13%)**	**14(2.99%)**
	**4**	**7(1.50%)**	**16(3.42%)**	**25(5.34%)**	***22(4.70%)***	***12(2.56%)***		**4**	**3(0.64%)**	**11(2.35%)**	**7(1.50%)**	***42(8.97%)***	***10(2.14%)***
	**5**	**4(0.85%)**	**6(1.28%)**	**11(2.35%)**	***37(7.91%)***	***54(11.54%)***		**5**	**0(%)**	**3(0.64%)**	**11(2.35%)**	***24(5.13%)***	***70(14.96%)***
**SI. (phi^2^ = 0.846, *p* < 0.001)**	**1**	***60(12.82%)***	***22(4.70%)***	**4(0.85%)**	**3(0.64%)**	**1(0.21%)**							
	**2**	***13(2.78%)***	***38(8.12%)***	**24(5.13%)**	**7(1.50%)**	**2(0.43%)**							
	**3**	**10(2.14%)**	**18(3.85%)**	**43(9.19%)**	**35(7.48%)**	**20(4.27%)**							
	**4**	**5(1.07%)**	**7(1.50%)**	**14(2.99%)**	***42(8.97%)***	***26(5.56%)***							
	**5**	**0(%)**	**4(0.85%)**	**5(1.07%)**	***11(2.35%)***	***54(11.54%)***							

*Cases in bold represent contrarian cases, while cases in italics represent the main effect. The sets of contrarian cases are counter to the main effect size (phi^2^ range from 0.05 to 1.04) at a significance level of 0.001. PE, perceived expectancy; FC, facilitating conditions; EE, effort expectancy; CV, cost value; SI, social influence.*
